# The Association Between Diet and Cardio-Metabolic Risk on Cognitive Performance: A Cross-Sectional Study of Middle-Aged Australian Adults

This article has been retracted.

**DOI:** 10.3389/fnut.2022.862475

**Published:** 2022-04-28

**Authors:** Sarah Gauci, Lauren M. Young, Lizanne Arnoldy, Andrew Scholey, David J. White, Annie-Claude Lassemillante, Denny Meyer, Andrew Pipingas

**Affiliations:** ^1^Centre of Human Psychopharmacology, Swinburne University, Melbourne, VIC, Australia; ^2^Food and Mood Centre, School of Medicine, Barwon Health, Institute for Mental and Physical Health and Clinical Translation, Deakin University, Geelong, VIC, Australia; ^3^Nutrition Dietetics and Food, School of Clinical Sciences, Monash University, Melbourne, VIC, Australia; ^4^Department of Health and Medical Sciences, Swinburne University, Melbourne, VIC, Australia; ^5^Department of Health Professions, Swinburne University, Melbourne, VIC, Australia; ^6^Department of Health Science and Biostatistics, Centre for Mental Health, Swinburne University, Melbourne, VIC, Australia

**Keywords:** diet, cognition, cardio-metabolic risk, mediterranean diet, MIND diet, DASH diet

## Abstract

Adherence to different dietary patterns has been linked to the development of cognitive decline; yet little is known about whether this relationship is present in middle age. The current study aimed to explore the relationship between different dietary patterns, cognitive performance, and potential cardio-metabolic mechanisms for this relationship. Participants were recruited using a diet screening tool to ensure that the cohort had a range of diet quality ranging from relatively poor to relatively healthy. In a sample of 141 middle-aged adults (age: M = 52.84 years, SD = 6.87 years), multiple 24 h diet recalls were collected and used to score adherence to the Mediterranean diet, dietary approaches to stop hypertension (DASH) diet, and Mediterranean–DASH diet intervention for neurodegenerative delay (MIND) diet. Metabolic risk was assessed using the metabolic syndrome severity score (MetSSS) and arterial stiffness. Cognitive performance was assessed using the Swinburne University Computerized Cognitive Assessment Battery (SUCCAB). Adherence to the MIND diet was significantly related to Stroop Processing domain (β = 0.19, *p* = 0.035). None of the dietary patterns were significantly related to MetSSS or arterial stiffness. However, adherence to the DASH diet was significantly associated with two cardio-metabolic measures including lower augmentation index (β = −0.17, *p* = 0.032) and lowered cholesterol (β = −0.18, *p* = 0.041). Interestingly, two cardio-metabolic risk factors were also associated with better cognitive performance: MetSSS (β = 0.21, *p* = 0.010) and waist circumference (β = 0.22, *p* = 0.020). Together these findings suggest that diet in middle age may be important for cognitive functioning and cardio-metabolic risk. However, more research is needed in the form of randomized controlled trials to confirm the direction of these relationships.

## Introduction

The global population is aging. By 2050, one in six people is expected to be over the age of 65 years (1). While longevity is a positive outcome of modern medicine, it also comes with an increased prevalence of age-associated cognitive decline and dementia. Critically, there are no effective pharmacological treatments that slow the progression of cognitive decline and dementia; there is a great need for effective prevention strategies and lifestyle interventions (2). To develop effective prevention strategies, there is a need to better understand the modifiable risk factors for these disorders, how to best mitigate them, and identify the optimal periods to intervene.

Over the last decade, there has also been a proliferation in research investigating the role that diet plays in the development of cognitive decline and, in turn, the development of dementia. The typical Western diet which is high in calories but low in nutritional value has been found to increase the risk of developing cognitive decline (3–5). The literature also proposes that nutrient-rich “healthy” diets are neuroprotective and may reduce the risk of developing cognitive decline and dementia (6–8). The diets with the most evidence for a favorable relationship with cognition include the Mediterranean diet (MedDiet), Dietary Approaches to Stop Hypertension (DASH) diet, and the Mediterranean–DASH Intervention for Neurodegenerative Delay (MIND) diet (5, 6). The direct mechanisms of how these diets improve cognitive functions are unknown. However, cardio-metabolic processes are suggested to be involved (9).

Cardiovascular disease is a well-established risk factor for cognitive decline and dementia (10–12). For example, hypertension, arterial stiffness, and coronary heart disease have all been found to increase the risk of developing dementia and cognitive decline (13–15). In addition to these cardiovascular health factors, metabolic syndrome (MetS) has also been linked to cognitive decline and an increased risk of dementia (16), however, this evidence is inconsistent, suggesting that more research is needed (17, 18). Recent research suggests that these health factors are particularly important in middle age for later-life cognitive performance (15, 19–22) and that midlife is a “critical period” to target the modifiable risk factors of cognitive decline and dementia (15, 23). A recent study of middle-aged Australian adults conducted by Young et al. (24) found that those with an optimal diet (assessed with a simple self-reported diet screening tool) have better Stroop Processing (a measure of executive functioning) compared with those with a suboptimal diet (24). Those with an optimal diet also had better nutritional status (higher Vitamin B6 and RBC folate and lower saturated fatty acids). These findings suggest that self-reported diet quality may impact cognition in middle age and this is reflected in nutrient status, however, the mechanisms underpinning this relationship are unclear. Furthermore, a better understanding of how more detailed dietary assessments and cardio-metabolic risk factors impact cognition in middle age is needed to provide evidence on when to target prevention strategies.

The current study aims to expand on the findings of Young et al. (24) by exploring the relationship between cognitive outcomes and dietary patterns, captured using detailed 24 h dietary assessments in a middle-aged cohort (24). We hypothesized that the more “healthy” dietary patterns (MedDiet, DASH, and MIND) would predict better cognitive performance in middle-aged adults. The study also aimed to explore the potential cardio-metabolic mechanisms by examining the relationship between diet, cardio-metabolic risk factors, and cognition.

## Materials and Methods

### Participants

This study utilized baseline data from the Memory and Attention Supplement Trial (MAST) cohort. The MAST RCT assessed the effects of a 12-week intervention of B vitamin-rich supplement on cognition and mood in healthy middle-aged adults (the results of the intervention will be published elsewhere). Data were collected at the Centre of Human Psychopharmacology at Swinburne University of Technology, Melbourne, Australia. All participants provided written informed consent to participate. The trial was approved by the Human Research Ethics Committee at Swinburne University of Technology and was registered with the Australian and New Zealand Clinical Trials Registry, and ClinicalTrials.gov, NCT03482063. The current article is an exploratory, cross-sectional study, using the baseline data from this clinical trial (*n* = 141), focusing on the relationship between different dietary patterns, cardio-metabolic risk factors, and cognitive performance before participants receiving the intervention (Figure 1).

**FIGURE 1:** Flowchart of participants included in the study and schedule of assessments used in this study.

All participants were recruited from the community using a combination of online advertising and posters. Participants were aged between 40 and 65 years. To recruit people with a range of diet quality, targeted advertising was used to recruit 50% of participants with an “optimal” diet and 50% of participants with a “suboptimal” diet. To achieve this goal, the diet quality of the participants was assessed before enrolment using the Diet Screening Tool (25). Participants scoring ≤ 59 were classified as having a “suboptimal” diet, whereas those scoring ≥ 60 were classified as an “optimal” (in this study, diet quality was used in the recruitment process, and more detailed dietary assessments were used in the current analyses). To be eligible to participate, participants needed to be free from any neurological conditions, cognitive impairment (MMSE score ≥ 25), and psychiatric disorders including depression (BDI < 20) and anxiety. Participants also had to be non smokers and free from any health conditions that would affect the absorption of food or significantly impact their cognitive performance (e.g., inflammatory bowel disease, coeliac disease, history of stroke, epilepsy, serious head trauma). Female participants were not able to participate if they were pregnant or lactating. Furthermore, participants were excluded if they were color blind or if they had uncontrolled hypertension (systolic > 160 mmHg and/or diastolic > 100 mmHg at rest). Participants were not permitted to take any medications, illicit drugs, or supplements that would impact their cognitive functioning for 4 weeks before testing.

### Cognitive Measures

Participants completed the Swinburne University Computerized Cognitive Assessment Battery (SUCCAB) (26). The battery was designed to assess cognitive performance and be sensitive to the changes associated with aging. It consists of eight tasks; Simple Reaction Time, Choice Reaction Time, Immediate/Delayed Recognition, Stroop Color–Word, Spatial Working Memory, and Contextual Memory (described in the following sections). Participants completed a short practice round before each task, all responses were recorded with a hand-held button box. Accuracy (% correct) and response time (ms) were calculated for each task. A performance measure was computed (accuracy/response time), to account for the speed-accuracy trade-off (27). A higher performance score indicates better cognitive performance on that task.

#### Simple Reaction Time

Participants were presented with the target of a single white square in the center of the screen. They were required to respond with a right button press with the appearance of the target, as quickly and as accurately as possible. There was a total of 30 targets, to avoid anticipation effects the targets were presented with a randomized inter-stimulus interval (ISI).

#### Choice Reaction Time

Participants were presented with either a blue triangle or red square. They needed to respond to the appearance of these shapes with a left (blue) or right (red) button press as quickly and as accurately as possible. Participants completed 20 trials.

#### Immediate/Delayed Recognition

Participants were shown a series of 40 abstract images, they were told to study these images. Each image was presented in the center of the screen for 3 s with no ISI. Once presented, a second series of 40 images were displayed including 20 from the original set and 20 that were new. Participants had to indicate if they recognized the image with a right (yes) or a left (no) button press. This task was then repeated at the end of the test battery, the remaining 20 images were presented with another 20 new images to assess delayed recognition.

#### Stroop Color–Word

Participants completed a congruent and incongruent Stroop task. There were four color words randomly presented to participants (blue, red, green, and yellow), these words were presented in either the congruent or incongruent color ink. Participants were asked to press the corresponding color button that matched the color of the ink, the words were presented in. These tasks were participant paced, once the participant selected an answer with a button press the next stimulus was presented.

#### Spatial Working Memory

Participants were presented with a 4 × 4 grid, six grid position containing white squares for 3 s. Participants were then presented with a blank grid, and four white squares were sequentially presented on the grid, participants were asked to respond with a yes or no button press to indicate if the square matched a position that was presented in the original pattern of white squares. There were a total of 14 trials, each trial was separated with a blank screen for 2 s. For each trial, two out of the four locations of white squares corresponded to the original grid position presented and two did not.

#### Contextual Memory

Participants were shown a series of 20 images of everyday objects, these were presented at either the top, bottom left, or right of the screen with no ISI. Once all presented the same, images were then presented in the center of the screen. Participants had to indicate the original location of the image with either a top, bottom, left, or right button press. As participants had to recall the spatial context of the image, this task assessed episodic memory.

#### Cognitive Domain Calculations

Performances on these eight tasks were combined into four cognitive domains (27). This was conducted to reduce the risk of Type I error. The four domains were Reaction and Decision Speed, Visual Processing, Spatial Working Memory, and Stroop Processing. These domains were computed using the method described by Kennedy et al. (27) whereby performance scores on each task were converted to Z scores to ensure each task contributed equal weight to their respective cognitive domain. Reaction and Decision Speed was calculated from an average of the performance on Simple Reaction Time and the Choice Reaction Time tasks. Visual Processing was derived from the average performance on the Immediate Recognition, Delayed Recognition, and Contextual Memory tasks. Spatial Working Memory was the average performance across the 14 Spatial Working Memory trials. Finally, Stroop Processing was calculated from the difference between performance on the Incongruent and Congruent Stroop tasks, this was a measure of inhibitory control.

### Dietary Assessment

Dietary data were collected using the Automated Self-Administered 24-Hour Dietary Assessment Tool (ASA24). Participants were required to enter all the food, drinks, and dietary supplements they consumed for 24-h, the assessment tool asks detailed questions about food form, preparation, portion size, and any additions to meals; this allows the food codes to be assigned to each item reported. The food and portion size options included in the recall were guided by the Australian Food, Supplement and Nutrient Database (AUSNUT) 2011-13 and data from the 2011–2013 Australian Health Survey. Nutrient intakes were calculated from the nutrient composition data from AUSNUT food and measure codes. Participants completed two diet recalls before their first testing session, an additional two recalls were completed in the 12 weeks after the first testing session. All available recalls (minimum of two and maximum of four) were used to calculate adherence to the DASH, MIND, and Mediterranean dietary patterns as this is more representative of habitual dietary intake (28). Participants who only completed two recalls (*n* = 21) and three recalls (*n* = 13) were also included in the analysis. Macronutrient content was compared between those with only two/three recalls to those with four and there was no significant difference in macros for energy, protein, fat, and carbohydrate consumption [*t*_(106)_ = 0.53, *p* = 0.599; *t*_(106)_ = −0.15, *p* = 884; *t*_(106)_ = 0.35, *p* = 0.726; *t*_(106)_ = −0.12, *p* = 0.902, respectively]. Therefore, participants with two or three recalls were also included in the analysis. In addition, sensitivity analysis was also conducted, removing participants with only two recalls and reported in the results for any significant findings. All dietary data were extracted from the ASA24, the AUSNUT 2011–2013 food items extract ranged from two to eight code items. Of these food items, those classified as mixed dishes were disaggregated using the AUSNUT 2011–2013 Food Recipe File. All dietary scoring was conducted by two researchers SG and LA. Dietary scores are described in Table 1, however, a more detailed scoring method will be published elsewhere.

**TABLE 1:** Dietary scores for MedDiet, DASH and MIND.

Food group	MedDiet			DASH			MIND		
	Item	Serves	Score	Item	Serves	Score	Item	Serves	Score
Oil and fat	Olive oil, % kcal from oil and fats	<50% ≥50% fats and oils	0 1	% kcal from fat	≥33 >30 to <33 ≤30	0 0.5 1	Olive oil	<50% ≥50% fats and oils	0 1
	Olive oil	<13.5 g ≥ 13.5 g	0 1	% kcal from saturated fatty acids	≥13 >10 to <13 ≤10	0 0.5 1			
Fruit and vegetables	Vegetables	<2 ≥2	0 1	Vegetables	<2 ≥2 to <4 ≥4	0 0.5 1	Green leafy vegetables	≤0.29 >0.29 to <0.86 ≥0.86	0 0.5 1
	Fruit	<3 ≥3	0 1	Fruits	<2 ≥2 to <4 ≥4	0 0.5 1	Other vegetables	<0.71 ≥0.71 to <1 ≥1	0 0.5 1
							Berries	<0.14 ≥0.14 to <0.29 ≥0.29	0 0.5 1
Meat	Red meat, hamburger, and meat products	>1 ≤1	0 1	Meats, poultry and fish	≥4 >2 to <4 ≤2	0 0.5 1	Red meat and products	≥1 ≥0.57 to <1 <0.57	0 0.5 1
	Chicken, % kcal from meat intake	≤50% >50%	0 1				Fish	<0. 033 ≥0.033 to <0.14 ≥0.14	0 0.5 1
	Fish and shellfish	<0.43 ≥0.43	0 1				Poultry	<0.14 ≥0.14 to <0.29 ≥0.29	0 0.5 1
Dairy	Butter, margarine and cream	>1 ≤1	0 1	Dairy	<1 ≥1 to <2 ≥2	0 0.5 1	Butter and margarine	>2 ≥1 to ≤ 2 <1	0 0.5 1
							Cheese	≥1 ≥0.14 to <1 <0.14	0 0.5 1
Nuts and legumes	Nuts	<0.43 ≥0.43	0 1	Nuts, seeds, and dry beans	<0.29 ≥0.29 to <0.57 ≥0.57	0 0.5 1	Nuts	<0.033 ≥0.033 to <0.71 ≥0.71	0 0.5 1
	Legumes	<0.43 ≥0.43	0 1				Beans	<0. 14 ≥0.14 to ≤0.43 >0.43	0 0.5 1
Grains				Total Grain intake	<5 ≥5 to <7 ≥7	0 0.5 1	Whole grains	<1 ≥1 to <3 ≥3	0 0.5 1
				Whole grain intake	<1 ≥1 to <2 ≥2	0 0.5 1			
Other	Sofrito	<0.29 ≥0.29	0 1	Sodium (mg/d)	>2,401 >1,500 to ≤2,401 ≤1,500	0 0.5 1			
Discretionary food	Commercial sweets or pastries	≥0.43 <0.43	0 1	Sweets	≥1.14 >0.71 to <1.14 ≤0.71	0 0.5 1	Pastries, sweets	≥1 ≥0.71 to <1 <0. 71	0 0.5 1
	Sweet carbonated beverages	≥1 <1	0 1				Fast/fried foods (times/ day)	≥0.57 ≥0.14 to <0.57 <0.14	0 0.5 1
Alcohol	Wine	<1 ≥1	0 1				Wine	>1 or 0 >0 to <1 1	0 0.5 1

*All in serves per day except those labeled differently. Definition of a serve was based on the original scoring of the diet, for serving sizes not reported in the original score, the USDA National Nutrient Database for Standard Reference dietary guidelines (2015–2020) was used to define a serve or the NIAA for alcohol (a more detailed description of scoring will be published elsewhere).*

#### Mediterranean Diet

The Mediterranean diet is a traditional dietary pattern commonly consumed by people living in the countries surrounding the Mediterranean Sea. It is high in fruits, vegetables, legumes, and grains; there is a moderate intake of oily fish and red wine; while having low consumption of red meat and processed foods, and olive oil is the main source of fat (29). To assess adherence to the Mediterranean diet, the 14-Item Mediterranean Diet Assessment Tool was used (30). Typically used in face-to-face assessments, the 14 items were scored after assessment using the data from the 24-h diet recalls. There is a total score of 14, with a higher number meaning greater adherence to the dietary pattern.

#### DASH Diet

The Dietary approaches to stop hypertension (DASH) diet was developed to help treat hypertension. It is high in fruits, vegetables, nuts, legumes, and whole grains (31). Adherence to the DASH diet was scored in accordance with the methods reported by Folsom et al. (31). Adherence was scored out of a total score of 11, with a higher score meaning greater adherence to the DASH diet.

#### MIND Diet

The Mediterranean DASH diet intervention for neurodegenerative delay (MIND) diet was created using evidence for the most neuroprotective components of both the Mediterranean diet and the DASH diet. The MIND has an emphasis on natural plant-based foods with limited intake of meat and food high in saturated fat. It also specifically highlights the consumption of berries and green leafy vegetables (32). Adherence to the MIND diet was scored in accordance with Morris et al.’s (32) and Mueller et al.’s (33) studies. There is a total score of 15, with a higher number meaning greater adherence to the dietary pattern.

### Cardio-Metabolic Risk Assessment

#### Cardiovascular Health Measures

Peripheral blood pressure was assessed using the SphygmoCor device (Model XCEL; AtCor Medical). For each participant, blood pressure was taken in the supine position from the left arm, with participants rested for 5 min before measurement. During this rest period, participants were instructed to relax and not talk as this may affect the reading. Blood pressure was assessed by taking three brachial pressure cuff assessments, the first recording was discarded, and the average was made using the second and third recordings. The brachial waveform was also analyzed using Pulse Wave Analysis (PWA), providing a non-invasive central blood pressure measurement with scores reported for central aortic systolic and diastolic blood pressure, pulse pressure (PP), augmentation pressure (AP), and augmentation index (AIx). PP is the difference between systolic and diastolic pressure.

The gold standard measurement of arterial stiffness is assessed as carotid–femoral-pulse wave velocity (cf-PWV). This was taken using the SphygmoCor device. Cf-PWV was calculated using a femoral cuff. This cuff measures the pressure pulse waveform from the femoral artery. While the participant is supine, the cuff was inflated to measure the pulse pressure waveform from the femoral artery, the research assistant concurrently measured the carotid waveform using a pressure tonometer probe (placed on the participant’s neck/carotid pulse). The distance between the two points (carotid and femoral) was measured to estimate the speed of the pressure pulse. cf-PWV is a well-validated method and is considered the gold standard for non-invasive arterial stiffness assessment (34). For each participant, two cf-PWV recordings were made, the recordings were then reviewed by SG and the recording with the lowest standard deviation was selected for analysis. For participants with two cf-PWV recordings with the same standard deviation, the score was averaged.

#### Blood Biomarkers

Biomarkers for lipids and glucose were assessed at the same visit as cardiovascular and cognitive assessments. Participants were required to come to the testing session fasted from 10 p.m. the night before. All blood samples were collected by a research nurse or venipuncture technician at the Centre for Human Psychopharmacology. The sample was collected into a serum separator tube (8.5 ml) with a clot activator (silicone and micronized silica) and was left to clot at room temperature for 30 min before being centrifuged for 10 min at 4,000 rpm. The sample was then couriered to Australian Clinical Labs where they were analyzed for full lipids and glucose.

#### Anthropomorphic Measures

Waist and hip circumferences were measured in accordance with the International Society for the Advancement of Kinanthropometry (ISAK) standards using anthropometric tape to the nearest 0.1 cm. BMI (weight in kilograms/height in m^2^) was computed from measured height and weight. Both height and weight were measured to the nearest 0.1 cm and 0.1 kg, respectively.

#### Metabolic Syndrome Severity Score

To assess the cardio-metabolic risk factor severity, the metabolic syndrome severity score (MetSSS) was used (35). The MetSSS is a standardized formula that calculates the overall risk or severity of cardio-metabolic syndrome. It uses the following measures to assess risk: waist circumference (cm), triglycerides (mmol/L), HDL cholesterol (mmol/L), Systolic BP (mmHg), diastolic BP (mmHg), and blood glucose (mmol/L).

### Statistical Analysis

All statistical analysis was conducted using IBM SPSS Statistics for Windows version 26 (IBM Corp., Armonk, NY, United States). For demographic and sample characteristic continuous variables were reported using means and standard deviations, while percentages were used to report categorical variables. To screen for outliers, Z scores were calculated for each variable and displayed in histogram form (*n* = 4 outliers treated as missing). Observations with values greatly disconnected from the data spread were considered outliers and were treated as missing. Accuracy operating below chance for cognitive tasks was recoded as missing and excluded from analysis for that task as this is indicative of not understanding the task (*n* = 2).

Cognition and cardio-metabolic variables (MetSSS, PWV, aortic and peripheral blood pressure, pulse pressure, augmentation pressure, augmentation index, glucose, total cholesterol, triglycerides, HDL cholesterol, and waist circumference) were then screened for normality and skewness by checking the skewness statistic (-1.96, 1.96). None of these outcomes were transformed.

The purpose of this statistical analysis was to explore the relationship between different dietary patterns (MedDiet, DASH, MIND), cardio-metabolic measures, and cognitive outcomes. Initially, Pearson’s correlations between the dietary pattern scores, cardio-metabolic variables, and cognitive domain scores were examined. Following this, separate hierarchical regression analyses were conducted with either dietary scores or cardio-metabolic risk factors (MetSSS and PWV) as the independent variable, with cognitive outcomes entered as the dependent variable while controlling for covariates. Covariates included age (in years), gender, years of education, and energy intake (kJ). Age, gender, and education were chosen as covariates as they are related to cognition and cognitive decline (36, 37). Energy (kJ) was included to account for differences in food intake.

For additional exploratory analysis, the components of the MetSSS and other cardio-vascular (aortic systolic blood pressure, aortic diastolic blood pressure, pulse pressure, augmentation pressure, augmentation index, glucose, total cholesterol, HDL cholesterol, and triglycerides) measures were analyzed for their relationship with cognition in additional hierarchical regression models. Finally, the relationship between dietary adherence and cardio-metabolic function was explored using hierarchical linear regression controlling for age and gender. As cognition was not an outcome for this analysis, education was not included as a covariate. All statistical significance was set at *p* < 0.0125 to allow for four cognition outcomes.

In the current study, a *post-hoc* power analysis was conducted using G*Power 3.1 (38), finding that when using nine variables in a model (four covariates, five independent variables), a 1.25% significance level to allow for four cognition outcomes, an estimated effect size of *f*^2^ = 0.15 and power of 0.80, a sample of 149 participants is required. Therefore, the current sample size is slightly underpowered.

## Results

### Sample Characteristics

Descriptive statistics for the sample are displayed in Table 2. There were 71 female participants (50.4%) and 70 male participants (49.3%). 35.5% of participants self-reported family history of cognitive disorder (yes/no). The majority of participants were low-to-moderate adherers to each of the dietary patterns, with a mean score of 5.34 out of a possible 14 for the MedDiet, 4.55 out of a possible 11 for the DASH diet, and 7.06 out of a possible 15 for the MIND diet.

**TABLE 2:** Characterization of the study sample for all participants.

	Mean	Standard Deviation	Minimum	Maximum	*n*
Age (years)	52.84	6.87	40.29	65.23	141
Education (years)	16.94	3.36	10.00	26.00	141
Body mass index	27.26	5.22	16.43	45.74	141
Waist circumference	95.91	14.77	71.00	137.50	140
MMSE	29.32	0.95	25.00	30.00	141
BDI-II	4.00	4.37	0.00	19.00	141

**Cardio-metabolic**					
Systolic BP	119.28	12.36	94.00	161.00	141
Diastolic BP	73.92	8.47	51.00	95.00	141
Aortic systolic BP	109.69	11.35	85.00	144.00	141
Aortic diastolic BP	74.76	8.54	52.00	96.00	141
Pulse pressure	34.93	6.18	23.00	55.00	141
Augmentation pressure	9.08	4.96	1.00	26.00	141
Augmentation index	25.38	11.53	2.00	63.00	141
PWV	9.47	1.26	6.30	13.50	132
MetSSS	1.41	1.47	0.00	6.49	137
Glucose mmol/L	5.04	0.54	4.10	6.90	134
Total cholesterol mmol/L	5.24	0.94	3.00	8.20	139
HDL cholesterol mmol/L	1.52	0.41	0.70	3.00	139
Triglycerides mmol/L	1.16	0.56	0.40	3.30	138

**Diet**					
Diet quality	62.10	13.00	35.00	93.00	141
DASH	4.55	1.63	1.5	8.5	141
MedDiet	5.34	1.71	2	10	141
MIND	7.06	1.98	2.5	13.0	141

**Ethnicity (*n*,%)**					
Caucasian	108	40.4			
Asian	10	7.1			
Other	23	16.3			

**Employment (*n*,%)**					
Full time	57	40.4			
Part time/casual	50	35.5			
Studying	2	1.4			
Retired	18	12.8			
Unemployed	14	9.9			

**Physical activity level (*n*,%)**					
Sedentary	1	0.7			
Insufficient	17	12.1			
Sufficient	123	87.2			

**Hormonal status (*n*,%)**					
Menstruating	25	35.2			
Peri-menopausal	8	11.3			
Post-menopausal	27	38.0			
Other^	11	15.5			

*^Other included post-hysterectomy or tubal ligation.*

### Correlations Between Variables

Initial analysis examined the correlations between the different dietary patterns and each cognitive domain score. The results from Spearman’s correlations are presented in Table 3.

**TABLE 3:** Correlations between dietary patterns and cognitive and cardio-metabolic outcome variables.

	MIND	DASH	R&DS	VP	SP	SWM	WC	Brachial SBP	Brachial DBP	Aortic SBP	Aortic DBP	PP	AP	AI	PWV	Glucose	Total cholesterol	Triglycerides	HDL	MetSSS
MedDiet	0.61**	0.45**	0.08	0.06	0.13	−0.08	−0.22**	−0.03	0.00	−0.04	0.01	−0.07	−0.07	−0.08	−0.09	−0.03	−0.04	−0.03	0.12	−0.10
MIND		0.55**	−0.05	−0.05	0.18*	−0.15	−0.28**	−0.05	−0.01	−0.04	−0.00	−0.07	−0.02	−0.01	−0.13	0.05	−0.03	−0.05	0.19*	−0.09
DASH			−0.09	0.00	0.06	0.02	−0.04	−0.04	−0.03	−0.05	−0.03	−0.05	−0.14^	−0.14^	−0.04	−0.08	−0.16^	_0.08	−0.04	−0.04
R&DS				0.47**	0.05	0.45**	0.13	0.02	0.00	0.00	0.00	0.01	−0.08	−0.09	0.01	0.05	−0.04	0.05	−0.11	0.11
VP			.		−0.08	0.50**	−0.05	0.00	−0.05	−0.03	−0.07	0.04	−0.04	−0.09	−0.08	−0.12	−0.01	−0.12	0.02	0.08
SP						−0.08	−0.12	−0.09	−0.14	−0.06	−0.15	0.10	0.18*	0.15^	−0.03	−0.00	−0.10	−0.11	0.09	−0.04
SWM							0.24**	0.05	−0.02	0.02	0.01	0.04	−0.11	−0.14	0.07	0.05	−0.04	0.05	−0.16^	0.24**

Pearson correlation coefficient, *p < 0.05, **p < 0.01, ^p < 0.10.

*MedDiet, Mediterranean Diet; MIND, Mediterranean-DASH Intervention for Neurodegenerative Delay; DASH, Dietary Approaches to Stop Hypertension; R&DS, Reaction and decision speed; VP, Visual processing; SP, Stroop Processing; SWM, Spatial working memory; SBP, Systolic blood pressure; DBP, Diastolic blood pressure; PP, Pulse pressure; AP, Augmentation pressure; PWV, pulse wave velocity; HDL, high-density lipoprotein cholesterol; MetSSS, Metabolic syndrome severity score; WC, waist circumference.*

There were significant positive correlations between each of the dietary pattern scores. Adherence to the MIND diet was also negatively correlated with waist circumference and HDL cholesterol. It was also positively correlated with Stroop Processing. Reaction and Decision Speed was positively correlated with Visual Processing and Spatial Working Memory. Visual Processing was significantly positively correlated with Spatial Working Memory. Stroop Processing was also positively correlated with Augmentation pressure. Finally, Spatial Working Memory was found to be positively correlated with waist circumferences and MetSSS.

### The Relationship Between Dietary Patterns and Cognitive Outcomes

Following the correlation analysis, separate hierarchical regressions were conducted, controlling for age, gender, education, and energy intake. The standardized regression coefficient for each analysis is shown in Table 4. Only the MIND diet was found to be significantly related to cognitive performance, specifically Stroop Processing [β = 0.19, *t*_(5,138)_ = 2.13, *p* = 0.035]. However, when removing participants with only two dietary recalls (*n* = 20) this was no longer significant [β = 0.14, *t*_(5,117)_ = 1.40, *p* = 0.165].

**TABLE 4:** Association of diet scores with cognitive performance, standardized coefficients beta, and adjusted *R*-Square.

	Reaction and decision speed		Visual processing		Stroop processing		Spatial working memory	
	β	*R* ^2^	β	*R* ^2^	β	*R* ^2^	β	*R* ^2^
MedDiet	0.08	0.03	0.03	0.06	0.13	0.01	−0.07	0.08
DASH	−0.10	0.04	0.03	0.06	0.06	0.00	0.04	0.07
MIND	−0.06	0.03	−0.12	0.07	0.19*	0.03	−0.13	0.09

Hierarchical regressions controlling for age, gender, education, and energy intake (kJ), *p < 0.05.

*MedDiet, Mediterranean Diet; MIND, Mediterranean-DASH Intervention for Neurodegenerative Delay; DASH, Dietary Approaches to Stop Hypertension.*

### The Relationship Between Cardio-Metabolic Measures and Cognitive Outcomes

To examine the associations between cardio-metabolic risk (MetSSS and PWV) and cognitive performance, hierarchical regression analyses were performed controlling for age, gender, and education. The regression coefficient and standard error for each analysis are shown in Table 5. As can be seen, a higher MetSSS significantly predicted better performance for SWM [β = 0.21, *t*_(4,136)_ = 2.61, *p* = 0.010]. PWV was not related to any of the cognitive outcomes.

**TABLE 5:** Association of cardio-metabolic measures with cognitive performance, standardized coefficients beta, and adjusted *R*-Square.

	Reaction and decision speed		Visual processing		Stroop processing		Spatial working memory	
	β	*R* ^2^	β	*R* ^2^	β	*R* ^2^	β	*R* ^2^
MetSSS	0.10	0.05	0.09	0.06	–0.02	–0.01	0.21*	0.11
PWV	0.07	0.04	0.05	0.06	–0.03	–0.02	0.16^∧^	0.10
**Exploratory analysis**								
Aortic SBP	0.03	0.03	0.02	0.05	–0.04	–0.02	0.08	0.08
Aortic DBP	0.02	0.03	0.01	0.05	–0.14	0.00	0.02	0.07
PP	0.03	0.03	0.05	0.05	0.13	–0.00	0.11	0.08
AP	–0.02	0.03	–0.08	0.06	0.19^*1^	0.04	0.00	0.07
AI	–0.03	0.03	–0.14	0.07	0.15	0.00	–0.03	0.07
Brachial SBP	0.04	0.03	0.06	0.05	–0.07	–0.01	0.09	0.08
Brachial DBP	0.02	0.03	0.00	0.05	–0.13	–0.00	0.03	0.07
Glucose	0.07	0.03	–0.05	0.05	0.04	–0.02	0.03	0.05
Total cholesterol	0.08	0.04	0.02	0.05	–0.10	–0.00	0.09	0.06
Triglycerides	0.00	0.04	–0.02	0.05	–0.08	–0.01	0.00	0.06
HDL	–0.07	0.05	–0.05	0.06	0.05	–0.01	–0.08	0.07
Waist circumference	0.13	0.04	0.04	0.05	–0.09	–0.01	0.22*	0.11

Hierarchical regressions controlling for age, gender, and education. *p < 0.05, ^p < 0.01. ^1^This was no longer significant when a multivariate outlier was removed.

*SBP, Systolic blood pressure; DBP, Diastolic blood pressure; PP, Pulse pressure; AP, Augmentation pressure; PWV, pulse wave velocity; HDL, high-density lipoprotein cholesterol; MetSSS, Metabolic syndrome severity score.*

For further exploratory analysis, the components that make up the MetSSS score, and other cardiovascular measures were examined in multiple hierarchical regressions. Waist circumference was found to be a significant predictor of Spatial Working Memory performance [β = 0.22, *t*_(4,139)_ = 2.36, *p* = 0.020]. Augmentation pressure was also found to predict Stroop Processing performance [β = 0.19, *t*_(4,138)_ = 2.06, *p* = 0.041]. However, when a multivariate outlier was removed, this was no longer significant [β = 0.16, *t*_(4,137)_ = 1.67, *p* = 0.097].

### The Relationship Between Dietary Patterns and Cardio-Metabolic Measures

To investigate the relationship between the different dietary patterns (MedDiet, DASH, and MIND) and the main cardio-metabolic outcomes (MetSSS and PWV), hierarchical regressions were completed controlling for age and gender. The results of these regressions are displayed in Table 6. Diet was not found to be significantly related to either MetS or PWV.

**TABLE 6:** Association of cardio-metabolic measures with dietary patterns, standardized coefficients beta, and adjusted R square.

	Main outcomes																		Exploratory analysis									
					MetSSS Components														Other cardiovascular measures									
	MetSSS		PWV		Brachial SBP		Brachial DBP		Glucose		Total cholesterol		Triglycerides		HDL		Waist circumference		Aortic SBP		Aortic DBP		Pulse pressure		AP		AI	
														
	β	*R* ^2^	β	*R* ^2^	β	*R* ^2^	β	*R* ^2^	β	*R* ^2^	β	*R* ^2^	β	*R* ^2^	β	*R* ^2^	β	*R* ^2^	β	*R* ^2^	β	*R* ^2^	B	*R* ^2^	β	*R* ^2^	β	*R* ^2^
MedDiet	−0.09	−0.01	−0.02	0.16	−0.02	0.07	0.02	0.04	0.01	0.12	−0.05	−0.02	−0.12	0.09	0.07	0.17	−0.11	0.23	−0.03	0.08	0.02	0.04	−0.08	0.07	−0.11	0.16	−0.12	0.16
DASH	−0.06	−0.01	−0.07	0.17	−0.08	0.08	−0.07	0.04	−0.15^	0.14	−0.18*	0.04	−0.11	0.09	−0.01	0.16	−0.09	0.23	−0.10	0.09	−0.07	0.05	−0.08	0.07	−0.15^^1^	0.16	−0.17*	0.17
MIND	−0.06	−0.01	−0.05	0.17	−0.01	0.07	0.04	0.04	−0.01	0.12	−0.04	−0.02	−0.09	0.08	0.09	0.17	−0.11	0.23	−0.02	0.08	0.04	0.04	−0.09	0.07	−0.10	0.16	−0.10	0.16

Hierarchical regressions controlling for age, gender, and energy. *p < 0.05, ^p < 0.01, ^1^after the removal of a multivariate outlier this is now significant.

*MedDiet, Mediterranean Diet; MIND, Mediterranean-DASH Intervention for Neurodegenerative Delay; DASH, Dietary Approaches to Stop Hypertension; SBP, Systolic blood pressure; DBP, Diastolic blood pressure; PP, Pulse pressure; AP, Augmentation pressure; PWV, pulse wave velocity; HDL, high-density lipoprotein cholesterol; MetSSS, Metabolic syndrome severity score.*

In addition, the relationships between the different dietary patterns and other cardio-metabolic outcomes were explored. Adherence to the DASH diet was associated with lower augmentation index [β = −0.17, *t*_(4,140)_ = −2.16, *p* = 0.032] and lower cholesterol [β = −0.18, *t*_(4,138)_ = −2.06, *p* = 0.041]. However, after the removal of a multivariate outlier adherence to the DASH diet was now significantly associated with lower augmentation pressure [β = −0.16, *t*_(4,139)_ = −2.07, *p* = 0.041]. After sensitivity analysis (removing participants with only two diet recalls) only cholesterol remained significant [β = −0.22, *t*_(4,118)_ = −2.31, *p* = 0.023], augmentation index [β = −0.15, *t*_(4,119)_ = −1.74, *p* = 0.085], and augmentation pressure [β = −0.15, *t*_(4,119)_ = −1.78, *p* = 0.077] were no longer significant.

## Discussion

The current study investigated the relationship between three dietary patterns (MedDiet, DASH, and MIND), cardio-metabolic risk factors, and cognitive performance in middle-aged adults. In this sample of Australian adults, greater adherence to the MIND diet was related to better cognitive performance on the Stroop Processing task. There were no significant relationships between adherence to the MedDiet and DASH dietary patterns and cognitive performance. The DASH dietary pattern was also found to predict two of the cardio-metabolic outcomes in this “healthy” cohort. Contrary to our hypotheses, higher values for both MetSSS and waist circumference were related to better spatial working memory.

To the authors’ knowledge, this is the first study to use a novel recruitment strategy targeting varied diet quality to explore the relationships between diet, cardio-metabolic risk, and cognitive outcomes in middle-aged adults. The significant finding between MIND diet adherence and greater Stroop Processing is consistent with past findings. In a recent study that assessed diet quality within the same sample, participants classified as having an “optimal” diet also had better Stoop processing (24). Hosking et al. (39) also found that adherence to the MIND diet and not the MedDiet was related to reduced incidence of cognitive impartment. This may be because the MIND diet was designed with brain and cognitive health in mind, choosing the aspects of both the MedDiet and DASH diet with the most evidence for neuroprotection (40). However, these findings need to be confirmed in a larger sample with participants who completed a minimum of 3–4 diet recalls. As the sensitivity analysis revealed that this relationship was no longer significant after removing participants with only two recalls (*n* = 20). Overall, the findings from the current study suggest that greater adherence to the MIND diet may be related to better cognitive performance.

Greater adherence to the DASH diet was found to predict favorable cardio-metabolic outcomes including lower augmentation index and total cholesterol. This is consistent with literature relating to the DASH diet, as it was originally designed to reduce hypertension and has been related to improved cardio-metabolic outcomes (31). Furthermore, these cardio-metabolic factors have been found to influence cognitive function and later-life risk of cognitive decline (11, 41). However, in the current study, metabolic risk (MetSSS) was found to be related to increased Spatial Working Memory performance. The relationship between increased metabolic risk and better cognitive performance is unexpected as metabolic syndrome in middle-aged women has been associated with accelerated cognitive decline (20). Furthermore, a greater number of metabolic syndrome components are related to worse cognitive performance for executive function and memory in middle-aged adults (19). However, after further exploration, the relationship between MetSSS and cognitive performance was found to be driven by waist circumference. While waist circumference has been related to poorer cognition in older women with type 2 diabetes (42), the current study was in middle-aged men and women free from diabetes. Furthermore, in older populations, lower body mass index has been related to increased cognitive decline, demonstrating that increased weight can play a protective role in some populations (43). The findings from this study suggest that in a sample of middle-aged healthy adults, waist circumference and higher metabolic risk may be protective of cognitive decline. Additionally, the longitudinal relationship between MetSSS, waist circumference, and cognitive outcomes needs to be further explored as the findings of the current study may be a by-product of the cross-sectional nature of the analysis. More research is needed to address if higher MetSSS and waist circumference in middle age are related to increased risk of cognitive decline later in life.

Another unexpected finding was the relationship between greater augmentation pressure and better Stroop Processing. As people age, their arteries begin to stiffen and this causes an increase in blood pressure and an increase in the pressure wave reflected to the heart with each heartbeat. Augmentation pressure is a measure of the increase in pressure that the wave reflection adds above systolic pressure (44). While it was predicted that increased blood pressure and arterial stiffness would be related to worse cognitive outcomes (15, 45), they were not related to cognition in the current study. A possible explanation for the current findings is that most of the participants in the current study had a healthy cardiovascular function and no one had uncontrolled hypertension. Moreover, previous research found that cardiovascular function and blood pressure do not have a linear relationship with cognition (15, 46). Therefore, when blood pressure is controlled, an increase in augmentation pressure may have a positive effect on cognition. However, there is growing evidence that worse cardio-metabolic function in middle age is related to worse cognitive function later in life (15, 20). Therefore, it is important to monitor cardio-metabolic health in middle age to ensure these risk factors are maintained in the healthy range. Taken in the context of the evidence reported in the literature, the findings of this study suggest that although there may not be a strong relationship between diet, metabolic risk, and cognition concurrently in middle age, these risk factors appear to be important for later life cognition and the development of cognitive decline.

The current study has some limitations that need to be taken into account when interpreting the findings. First, this study is cross-sectional in nature—current dietary intake may not represent habitual dietary intake and this may therefore explain the lack of a significant relationship between the dietary patterns examined and the cognition. Second, although 24 h diet recalls provide detailed dietary information, they are still prone to reporting errors. Biochemical markers of diet quality are more accurate as they take into account what is absorbed into the body and can account for social desirability biases (24, 47). Finally, many statistical comparisons have been made in this current study, this means that it is vulnerable to Type 1 error, and no corrections for multiple comparisons were made. Therefore, the findings should be interpreted with caution.

While there are several limitations, there are also many strengths. First, there are a limited number of published studies investigating the concurrent relationship between diet and cognition in middle age (5). This study addresses this gap in the literature as the age of participants recruited were healthy middle aged (40–65 years). Second, the cognitive outcomes utilized in this study are sensitive to the cognitive domains that decline with age. This is particularly important in a healthy population free from cognitive decline. Finally, another important strength of this study was the recruitment technique used. By targeting 50% of participants with optimal diets and 50% with “sub optimal” diets, it enabled a broader range of participants to be recruited (although the overall *n* was relatively low), allowing for greater variability in diet quality than is typical for such studies (24).

## Conclusion

The present study examined the relationship between adherence to the MedDiet, DASH, and MIND diet, cardio-metabolic risk, and cognitive performance in middle-aged Australian adults. Only the MIND diet was significantly related to cognition (better Stroop Processing). There were, however, significant relationships between adherence to the DASH diet and cardio-metabolic factors. These findings suggest that in a healthy sample of adults, the MIND diet, which was developed using nutrition evidence for brain health, may be related to better cognitive performance. However, the DASH diet was favorably related to cardio-metabolic risk factors and therefore may have an indirect impact on cognition later in life. Unexpectedly, MetSSS and waist circumference were found to be related to greater Spatial Working Memory performance, and augmentation pressure was related to better Stroop Processing. These findings suggest that the relationship between cardio-metabolic risk and cognition may not be linear. Overall, the current literature suggests that diet in middle age may be important for cognition and cardio-metabolic health. However, more research including longitudinal and prospective studies as well as randomized controlled trials are needed to confirm this.

## Data Availability Statement

The data analyzed in this study is subject to the following licenses/restrictions: Need ethical clearance to access data. Requests to access these datasets should be directed to apipingas@swin.edu.au.

## Ethics Statement

This study involved human participants was reviewed and approved by Swinburne University Human Research Ethics Committee (SUHREC Project No. 2017/269). The participants provided their written informed consent to participate in this study.

## Author Contributions

LY and SG were largely responsible for recruitment and data collection. SG drafted the manuscript. SG and LA scored the dietary patterns. All authors conceived the study, had significant input into design, participated in revision of the manuscript, contributed to the article, and approved the submitted version.

## Conflict of Interest

AS, DW, and AP have received research funding honoraria and conference support and consultancy from the nutrition industry. AP has previously served as a member of the Scientific Advisory Panel for Swisse Wellness Pty Ltd. The remaining authors declare that the research was conducted in the absence of any commercial or financial relationships that could be construed as a potential conflict of interest.

## Publisher’s Note

All claims expressed in this article are solely those of the authors and do not necessarily represent those of their affiliated organizations, or those of the publisher, the editors and the reviewers. Any product that may be evaluated in this article, or claim that may be made by its manufacturer, is not guaranteed or endorsed by the publisher.
